The article "RNA interference targeting human integrin α6 suppresses the metastasis potential of hepatocellular carcinoma cells" was published in 2013. Journal: Eur J Med Res.

# RNA interference targeting human integrin α6 suppresses the metastasis potential of hepatocellular carcinoma cells

**DOI:** 10.1186/2047-783X-18-52

**Published:** 2013-12-04

**Authors:** Guannan Lv, Tianjing Lv, Shifeng Qiao, Wei Li, Weiran Gao, Xiaohui Zhao, Jikun Wang

**Affiliations:** 1 The First Affiliated Hospital of Liaoning Medical College, Jinzhou 121001, China; 2 Institute of Urology, Peking University First Hospital, Peking University, Beijing 100034, China

**Keywords:** Hepatocellular carcinoma, integrin α6, Short hairpin RNA, Metastasis

## Abstract

**Background:**

Increased metastasis has been proved to be associated with a poor prognosis for hepatocellular carcinoma (HCC). There are higher-level expressions of integrin α6 in the tissues of HCC patients with a higher fatality rate. The aim of this study is to investigate the effect of short hairpin RNA (shRNA) silencing integrin α6 expression on the proliferation and metastasis in HCC cell lines.

**Methods:**

Two human HCC cell lines, HepG2 and Bel-7402 were transfected with shRNA targeting human integrin α6. Protein and mRNA expression level were determined by western blot and real-time quantitative reverse transcription-polymerase chain reaction (qRT-PCR) to detect the transfected efficacy. The metastasis potential of HCC cells was evaluated by their proliferation, adhesion and invasion abilities. Cell proliferation was measured by MTT assay. Adhesion ability was measured by adhesion and spreading assays. The expression of matrix metalloproteinases (MMPs) was measured by qRT-PCR. The potential of invasion was measured by qRT-PCR and Transwell chamber assay. PI3K inhibitor LY294002 was used to explore the signal pathways of integrin α6 in HCC cells.

**Results:**

Western blot and qRT-PCR detection showed that over 75% of integrin α6 expression in HCC cells was through knockdown by shRNA. Proliferation, adhesion, spreading and invasion of HepG2 and Bel-7402 cells were dramatically decreased in cells transfected with shRNA compared to the control cells. P-ERK and p-AKT were reduced by shRNA targeting integrin α6 and PI3K inhibitor LY294002.

**Conclusion:**

Knockdown integrin α6 can inhibit the proliferation and metastasis of HCC cells through PI3K/ARK and MAPK/ERK signal pathways by shRNA *in vitro*. Integrin α6 can mediate the metastasis potential, and can be used as a candidate target for therapy in HCC resulting in improved patients’ survival.

## Background

Hepatocellular carcinoma (HCC) is a highly lethal cancer with a poor prognosis. The occurrence of HCC has recently shown a worldwide increase [1], mainly because of its high metastasis potential [2].

Integrins are heterodimeric transmembrane receptors composed of non-covalently associated α and β subunits. At least 18 α and 8 β subunits have been identified so far, generating more than 24 members of the integrin family. Increasing evidence suggests that integrins are the most important receptors for cell metastasis [3]. Recently, it has been reported in many researches that integrin α6β1 and α6β4 were associated with metastasis of HCC [4,5] and patients with high levels of expression of integrin α6β1 have a poorer prognosis [4,6]. Higher levels of expression of integrin α6β4 in patients is associated with increased invasive potential of HCC, as well as a higher fatality rate [5,7]. Integrin α6β1, as an important kind of cell surface receptor, can mediate the adhesion between HCC cells and extracellular matrix (ECM) [8,9]. Owens *et al*. [10] demonstrates that integrin α6β4 could regulate the migration and invasion of laminin (LN) to stimulate the metastasis potential of HCC.

The article "RNA interference targeting human integrin α6 suppresses the metastasis potential of hepatocellular carcinoma cells" was published in 2013. Journal: Eur J Med Res.

However, few research studies have focused on the single action of integrin α6 alone in the progression of HCC metastasis. Furthermore, the metastatic mechanisms under high levels of expression of integrin α6 are still unclear. A better understanding of the molecular mechanisms underlying integrin α6 affecting HCC metastasis may facilitate the development of targeted therapy.

In the current study, in order to explore the effect of integrin α6 in the process of HCC metastasis without the influence of β subunits and the molecular mechanisms involved, two human HCC cell line, HepG2 and Bel-7402 were transfected with short hairpin RNA (shRNA) targeting human integrin α6. The metastasis potential of HCC cells was evaluated by proliferation, adhesion and invasion abilities. PI3K inhibitor LY294002 was also used to explore the signal pathway of integrin α6 in HCC cells.

## Methods

### Cell culture and plasmids preparation

Two hepatocellular cell lines, HepG2 and Bel-7402 were purchased from the Chinese Academy of Medical Science (Beijing, China). All cells were cultured in RPMI 1640 (Life Technologies Corporation, 5791 Van Allen Way, Carlsbad, CA 92008, US) with 10% FBS, 200 μg/ml penicillin and streptomycin at 37°C in 5% CO_2_. Integrin α6 shRNA plasmids (sc-43129-sh) were constructed and synthesized by Santa Cruz Biotechnology, Inc., CA, USA. Plasmids containing puromycin resistance genes were used for the selection of cells stably expressing shRNA. Control shRNA plasmids (sc-108065), each encoding a scrambled shRNA sequence that will not lead to the specific degradation of any known cellular mRNA, were also purchased from Santa Cruz Biotechnology, Inc., CA, USA.

### Cell transfection and clone selection

Integrin α6 shRNA plasmids or control shRNA plasmids were transfected into HepG2 and Bel-7402 cells respectively, according to the manufacturer's instructions with slight modification. Briefly, in a 24-well tissue culture plate, cells were grown to approaching up to 85% to 90% confluence in RPMI 1640 with 10% FBS. The medium was aspirated 24 hours before transfection, and replaced with DMEM. Lipofectamine 2000 (Invitrogen, Carlsbad, CA, USA) 0.5 μl and plasmids 0.02 μg were added in each well and incubated for six hours. After that, cells were cultured in RPMI 1640 with 20% FBS, 400 μg/ml penicillin and streptomycin for 18 hours. After replacing the media with fresh normal growth medium, cells were incubated for an additional 24 hours. Three days later, stable transfectant clones were isolated with 1.6 μg/ml and 2 μg/ml puromycin (Santa Cruz Biotechnology, Inc., CA, USA) in HepG2 and Bel-7402 respectively.

The article "RNA interference targeting human integrin α6 suppresses the metastasis potential of hepatocellular carcinoma cells" was published in 2013. Journal: Eur J Med Res.

### RNA extraction and qRT-PCR assays

Briefly, 2 μg total RNA was used to synthesize first-strand cDNA. Amplification and detection were performed using the ABI Prism 7500 Fast Real-time System (Applied Biosystems, Foster City, California, USA) starting with 1 μl cDNA and TransStart Top Green qPCR SuperMix (TransGen Biotech, Beijing, China). Glyceraldehyde 3-phosphate dehydrogenase (GAPDH) was used as internal standard.

Primers sequences for integrin α6, matrix metalloproteinase (MMP)-2, MMP-9 and GAPDH were as follows:

Integrin α6: 5’-TCCCTGAACCTAACGGAGT-3’ and 5’-ATGTCCAAGTAGTTC AGTT-3’;

MMPs-2: 5’-GCGACAAGAAGTATGGCTT-3’ and 5’-TGCCAAGGTCAATGT CAGG-3’;

MMPs-9: 5’-AGTTCCCGGAGTGAGTTGA-3’ and 5’-CTCCACTCCTCCCTT TCCT-3’;

GAPDH: 5’-GGCATCCTGGGCTACACTG-3’ and 5’-GTGGTCGTTGAGGGCAATG-3’.

The relative expression of integrin α6, MMP-2 and MMP-9 mRNA was analyzed by the comparative cycle threshold (Ct) method. All experiments were performed in triplicate.

### Western blot assays

Cells (1 × 10^6^) were washed with PBS twice and lysed with 1 ml RIPA lysis buffer supplemented with 40 mmol/L NaF, 100 μmol/L Na_3_VO_4_, and 1 μl Complete Protease Inhibitor (KeyGen Biotech Co. Ltd, Nanjing, China) for 30 minutes on ice. After removing the insoluble material by 12,000 × g centrifugation for 30 minutes at 4°C, the supernatants were collected, boiled in 1 × sodium dodecyl sulfate sample buffer for five minutes. Subsequent immunoblots were probed with the appropriate antibody and detected by Gel Imaging System G: BOX (Gene Company Limited, Cambridge, UK). Monoclonal rabbit anti-human CD49f (1:100, Abgent, San Diego, CA, USA), rabbit anti-human AKT (1:200); rabbit anti-human p-AKT (1:200); rabbit anti-human ERK (1:200); and rabbit anti-human p-ERK (1:200); antibody (these last four supplied by Santa Cruz Biotechnology, Inc., CA, USA), were used to detect the expression of integrin α6, AKT, p-AKT, ERK, and p-ERK respectively. GAPDH (1:500; Santa Cruz Biotechnology, Inc., CA, USA) was used as internal control.

The article "RNA interference targeting human integrin α6 suppresses the metastasis potential of hepatocellular carcinoma cells" was published in 2013. Journal: Eur J Med Res.

### Cell proliferation assays

Cell proliferation was determined by MTT assay in accordance with other studies [11]. Briefly, 2 μg/cm^2^ of LN (Sigma, St. Louis, MO, USA) was placed on a ten-dish plate and allowed to solidify at 37°C for two hours. The other wells were coated with 2 μg/cm^2^ of fibronectin (FN) (Sigma, St. Louis, MO, USA) as control. After washing each well twice with PBS, 8 × 10^3^ cells were incubated in 96-well plates with DMEM containing 10% FBS at 37°C in 5% CO_2_ for 48 hours. MTT (10 μl) was added to each well and four hours later, the media was aspirated and 100 μl dimethyl sulfoxide (DMSO) was added. The assay was quantified in a Multimode Microplate Reader-Varioskan Flash (Thermo Electron Corporation, Waltham, MA, USA) at 490 nm. All experiments were repeated in at least quadruplicate.

### In vitro adhesion assay

LN or FN was coated in 96-well plates according to the method described above [12]. In total, 8 × 10^3^ cells suspended in DMEM were cultured at 37°C in 5% CO_2_ for 30 minutes. After being washed with DMEM three times, acid phosphatase substrate consisting of 0.1 mol/l sodium acetate buffer (pH 5.5), 0.1% Triton X-100 (10 mmol/L), and nitrophenylphosphate 100 μl were added to each well. The cells were cultured at 37°C for two hours, then 1 mol/L NaOH 10 μl was added to each well to stop the reaction. The adhesion assay was quantified in a Multimode Microplate Reader-Varioskan Flash (Thermo, Electron Corporation, Waltham, MA, USA) at 405 nm. All the results were obtained from at least three independent experiments.

### In vitro spreading assay

LN was coated in 96-well plates according to the method described above. In total, 8 × 10^3^ cells suspended in DMEM were cultured at 37°C at 5% CO_2_ for 150 minutes. Then, a light microscope (×200) was used to determine the spreading assay. In this experiment, spreading cells were counted respectively in three distinct visions.

### LN invasion assay

The upper part of the Transwell chambers coated with LN was used as a basement membrane (BM) according to the way described above. Fibronectin (FN) was used as control. Cells (1 × 10^5^) suspended in DMEM containing 0.1% FBS were plated in the upper part to make contact with the BM. BSA (0.05%) in DMEM with 10% FBS was placed in the lower chamber, to act as chemoattractants. Cell invasion was determined by crystal violet dissolution assay after incubation at 37°C in 5% CO_2_ for 48 hours; the invaded cells were numerated under a light microscope (×400). In this experiment, invaded cells were counted in three distinct microscopic fields respectively.

The article "RNA interference targeting human integrin α6 suppresses the metastasis potential of hepatocellular carcinoma cells" was published in 2013. Journal: Eur J Med Res.

### The signal pathways assay

LN or FN was coated in 24-well plates according to the method described above. Cells (1.5 × 10^6^), serum-starved for 48 hours, were allowed to adhere to the LN or FN and incubated at 37°C in 5% CO_2_ for two hours. In order to demonstrate the PI3K/AKT and MAPK/ERK signal pathways, which are necessary for the reaction between HCC cells and LN, PI3K inhibitor LY294002 was used one hour before HepG2 cells were cultured in plates coated with 2 μg/cm^2^ of LN. DMSO was used as control. Protein and mRNA were extracted and analyzed as described in the western blot assay and real-time quantitative reverse transcription-polymerase chain reaction (qRT-PCR) assay.

### Statistical analysis

Statistical analysis was performed with SPSS 15.0 for Windows (Chicago, IL, USA). Values are expressed as the mean ± standard deviation. The student *t-*test was used for comparison between groups. *P* < 0.05 was considered statistically significant.

## Results

### The stable transfection of integrin α6-shRNA plasmid dramatically down-regulated the expression of integrin α6

As shown in Figure 1, in the western blot assay, compared with the control group, the protein grayscale value of integrin α6 reduced remarkably in the HepG2-shRNA-integrin α6 cells (Figure 1A). In the qRT-PCR assays, compared with the control group, the relative integrin α6 mRNA reduced remarkably (*P* < 0.05) (Figure 1B). About 75% of integrin α6 was from knockdown by shRNA. The same result can be found in Bel-7402 cells (*P* < 0.001).

**Figure 1:** **HepG2 and Bel-7402 cells were infected with integrin α6 short hairpin RNA (shRNA) plasmids and control shRNA plasmids respectively.** Stable transfectant clones were picked up by puromycin. Integrin α6 expression levels remarkably reduced. **(A)** Western blot assays yielded the expression level of integrin α6 on protein level in HepG2 and Bel-7402 cell lines. **(B)** The qRT-PCR assays showed the expression level of integrin α6 on mRNA level in HepG2 and Bel-7402 cell lines. *P < 0.05; ***P < 0.001 compared with control group.

The results demonstrated that the expression level of integrin α6 was dramatically down-regulated after stable transfection at both protein and RNA level with significant statistical difference.

### Lower integrin α6 expression caused decreased proliferation of HCC cells on LN

As shown in Figure 2, a lower level of integrin α6 caused decreased proliferation of HCC cells on LN. This suggested that the proliferation of HCC cells was associated with the expression level of integrin α6 reacting with LN.

The article "RNA interference targeting human integrin α6 suppresses the metastasis potential of hepatocellular carcinoma cells" was published in 2013. Journal: Eur J Med Res.

**Figure 2:** **Cells were incubated in 96-well plates coated with laminin (LN) or fibronectin (FN) respectively for 48 hours.** The MTT assays showed that the lower-level expression of integrin α6 caused decreased proliferation of HCC cells with significant statistical difference (*P* < 0.05) in the cells incubated on LN, while the cells incubated on FN did not show any statistically significant effect (*P* > 0.05). *P < 0.05, ****P < 0.0001 compared with control group.

### Lower integrin α6 expression caused decreased invasion potential of HCC cells

To specifically address the importance role of integrin α6 in the invasion of HCC cells, we performed the Transwell experiments coated with LN or FN. We found that cells expressing lower-level integrin α6 showed a lower invasion potential (Figure 3). A total of 91.0 ± 1.33 HepG2-control shRNA cells crossing LN, compared to 8.67 ± 1.56 in the HepG2-integrin α6 shRNA cells (*P* < 0.0001) (Figure 3D). Furthermore, the number of HepG2-control shRNA cells crossing FN (75.0 ± 2.67) was significantly less than the cells crossing LN (*P* = 0.0034) (Figure 3D). These results indicated that lower-level expression of integrin α6 caused decreased invasion potential for HCC cells, and LN can increase invasion potential of HCC cells with high integrin α6 levels.

**Figure 3:** **Cells were cultured in Transwell chambers with the upper part coated with laminin (LN) or fibronectin (FN) respectively for 48 hours.** The invaded cells were numerated under a light microscope (×400). **(A)** HepG2 infected by control shRNA plasmids invaded LN. **(B)** HepG2 cells infected by control shRNA plasmids invaded FN. **(C)** HepG2 cells infected by integrin α6 shRNA plasmids invaded LN. HepG2 had a decreased invasion potential after the knockdown of integrin α6 with significant statistical difference (*P* < 0.0001). It also proved that LN can increase invasion potential of HepG2 (*P* < 0.05).

### Lower integrin α6 expression reduced invasion potential of HCC cells through the down-regulation of adhesion ability, spreading ability and secretion of MMPs

It has been mentioned above that adhesion and spreading is the first step of the model for tumor metastasis reported by Liotta *et al*., so we performed adhesion and spreading assays *in vitro*. These yielded results showing that the adhesion ability reduced remarkably in the HCC cells with lower-level expression of integrin α6 (*P* < 0.0001) (Figure 4A). On spreading, the results showed that HepG2 cells with lower level of integrin α6 had a lower rate of spreading (2.4% in the HepG2-shRNA-integrin α6 and 94% in the HepG2) (Figure 4B). The qRT-PCR assay was used to detect the relative integrin MMP-2 and MMP-9 levels. Compared with control group, the relative MMP-2 and MMP-9 mRNA reduced remarkably (*P* < 0.01) (Figure 4C, D). Thus, the down-regulation of MMP-2 and MMP-9 secretion, adhesion and spreading ability may cause the low invasion potential of HCC cells.

The article "RNA interference targeting human integrin α6 suppresses the metastasis potential of hepatocellular carcinoma cells" was published in 2013. Journal: Eur J Med Res.

**Figure 4:** **Cells were cultured in 96-well plates coated with laminin (LN) or fibronectin (FN) respectively for 30 minutes and then cultured with acid phosphatase substrate at 37°C.** The reaction was stopped two hours later. **(A)** The adhesion assays showed that lower-level integrin α6 reduced the adhesion of HCC cells with significantly statistical difference (*P* < 0.0001) in the cells incubated with LN, while the cells incubated with FN did not show any significant effect (*P* > 0.05). **(B)** Cells cultured in 96-well plates were coated with LN for 150 minutes. The spreading cells were numerated under a light microscope (×200). HepG2 cells with lower level of integrin α6 had a lower spreading rate. **(C)** The qRT-PCR assay showed that MMP-2 expression reduced significantly at mRNA level (*P* < 0.01). **(D)** The qRT-PCR assay showed that MMP-9 expression reduced significantly at RNA level (*P* < 0.01). *P < 0.05, **P < 0.01, ****P < 0.0001 compared with control.

### Integrin α6 reacting with LN induced the hyperactivation of PI3K/AKT and MAPK/ERK signal pathways

As shown in Figure 5, compared with the control group, the protein grayscale value of p-ERK, p-AKT was dramatically reduced in HepG2 cells transfected with integrin α6 shRNA plasmids compared with control shRNA plasmids (Figure 5A, B). As revealed in Figure 5C, LY294002 decreased both the expression of p-ERK and p-AKT, but had no influence on the expression of ERK and AKT. The proliferation of HepG2 cells was remarkably decreased after being inhibited by PI3K (*P* < 0.05) (Figure 5D). In Transwell assays, 38.33 ± 3.78 cells crossed LN in the HepG2/LY294002 group, while 64.0 ± 2.67 cells in the HepG2/DMSO group and 72.33 ± 3.11 cells in HepG2 group (*P* < 0.05) (Figure 5E) crossed LN. These results demonstrated that the reacting of integrin α6 with LN induced the hyperactivation of PI3K/AKT and MAPK/ERK signal pathways.

**Figure 5:** **Expression levels determination of PI3K/AKT and MAPK/ERK. (A)** Western blot assay revealed the expression level of p-ERK was lower in HepG2 and Bel-7402 cells transfected with integrin α6 short hairpin RNA (shRNA) plasmids, while the expression of ERK remained unchanged. Cells transfected with control shRNA plasmids show no difference on p-ERK and ERK expression. **(B)** Western blot assay revealed the expression of p-AKT was lower in HepG2 and Bel-7402 cells transfected with integrin α6 shRNA plasmids, while the expression level of AKT remained unchanged. Cells transfected with control shRNA plasmids show no difference in p-AKT and AKT expression. **(C)** Western blot assay showed that PI3K inhibitor LY294002 reduced the expression of both p-AKT and p-ERK. **(D)** MTT assay showed that the proliferation of HepG2 cells cultured with LY294002 was dramatically reduced (*P* < 0.05). **(E)** Transwell assay showed that the invasion potential of HepG2 cells cultured with LY294002 was dramatically reduced (*P* < 0.05). *P < 0.05 compared with control.

The article "RNA interference targeting human integrin α6 suppresses the metastasis potential of hepatocellular carcinoma cells" was published in 2013. Journal: Eur J Med Res.

## Discussion

Metastatic recurrence is the main obstacle to the improvement of treatment efficacy for HCC [13], and heterodimeric transmembrane protein generated by integrin α6 subunits is suggested to be associated with metastasis potential of HCC. In this study, we used LN, the important structural component of ECM and integrin α6 ligand, as a model molecule and applied several assays to determine the importance of integrin α6 in the metastasis of HCC cells. In order to make the results more objective, the integrin α6 shRNA was used to silence the expression of integrin α6 of two HCC cell lines at RNA level. Western blot and qRT-PCR detection showed that over 75% of integrin α6 expression in HCC cells was through knockdown by shRNA.

Tumor metastasis is a multi-step process involving various molecules, pathways and organs. This process mainly includes the following steps before invasion to form micrometastases in the metastatic site: the detachment of tumor cells from a primary tumor, invasion through the stromal tissues, intravasation into the blood/lymph vessels, arrest in capillary bed followed by extravasation and local crawling [14].

Based on the results of our assays, lower-level integrinα6 expression down-regulated the secretion of matrix metalloproteinases (MMPs), the adhesion force between HCC cells and LN, the spreading ability on the LN, as well as the invasion potential of HCC cells. p-ERK and p-AKT were reduced by shRNA targeting integrin α6 and PI3K inhibitor LY294002. LN could stimulate the MMPs secreted by HCC and thus was associated with a more metastatic phenotype of HCC cells [15]. The phosphorylation level of ERK and AKT (p-ERK and p-AKT), which has been reported to be increased after combining integrin α6 with LN [16,17], is associated with a low survival rate for HCC patients [17]. Furthermore, influencing factors increase the secretion of MMP-9 through the activation of the MAPK/ERK signal pathway, which is conducive with HCC metastasis [18]. The same results have been found in the PI3K/AKT signal by Chen *et al*. [19].

The article "RNA interference targeting human integrin α6 suppresses the metastasis potential of hepatocellular carcinoma cells" was published in 2013. Journal: Eur J Med Res.

A model for tumor metastasis reported by Liotta *et al*. [20] in the early 1980s contributes in large part to the metastatic process. The model mentions that there are three stages for the complicated interactions between tumor cells and ECM: the adhesion of tumor cells to the ECM, secretion of proteolytic enzymes, such as MMPs, directly by the tumor cells or indirectly by the host cells as a response to the presence of tumor cells, and finally, cell movement by chemotaxis or haptotaxis. Although most integrin family members recognize more than one ECM protein, integrin α6 is a ligand with specificity for LN [21,22]. The signal pathways, MAPK/ERK and PI3K/AKT have been proved to be necessary for HCC metastasis [19,23]. Thus, we can hypothesize that the combination of integrin α6 with LN could influence the HCC metastasis by affecting cell adhesion and migration, and reduced expression level of integrin α6 may cause low potential of HCC metastasis through the activation of MAPK/ERK and PI3K/AKT signal pathways. There also exist cross-talk between the two signaling pathways activated by LN [18,19]. Integrin α6 contributes to the regulation of interaction between HCC cells and LN through PI3K/AKT and MAPK/ERK signaling pathways which are shown to be essential for the metastasis of HCC [6].

## Conclusions

Down-regulation of integrin α6 could decrease the potential of HCC metastasis through reducing the interaction between HCC and LN. This study showed that over-expression of integrin α6 in HCC is a strong indicator for more aggressive tumors and poorer clinical outcome. All the currently available therapies for HCC are mainly oriented towards removing or destroying the tumors, whereas few therapies aim at blocking the process of HCC metastasis [24]. This study would help us to understand the metastatic process of HCC better and develop targeted molecular therapy to improve patients’ survival.

## Abbreviations

HCC: Hepatocellular carcinoma; shRNA: Short hairpin RNA; qRT-PCR: Real-time quantitative reverse transcription-polymerase chain reaction; MMPs: Matrix metalloproteinases; ECM: Extracellular matrix; LN: Laminin; Ct: Cycle threshold; DMSO: Dimethyl sulfoxide; FN: Fibronectin.

## Competing interests

The authors declare that they have no competing interests.

## Authors’ contributions

GNL conducted experiments, prepared manuscript and analyzed data. TJLand SFQ performed experiments, revised manuscript and analyzed data. WL performed experiments. WRG performed experiments. XHZ erformed experiments. JKW designed experiments and gave final approval of manuscript. All authors read and approved the final manuscript.
